# Nuciferine inhibits the progression of glioblastoma by suppressing the SOX2-AKT/STAT3-Slug signaling pathway

This article has been retracted.

**DOI:** 10.1186/s13046-019-1134-y

**Published:** 2019-03-29

**Authors:** Zizhuo Li, Yaodong Chen, Tingting An, Pengfei Liu, Jiyuan Zhu, Haichao Yang, Wei Zhang, Tianxiu Dong, Jian Jiang, Yu Zhang, Maitao Jiang, Xiuhua Yang

**Affiliations:** 1 Department of Abdominal Ultrasound, The First Affiliated Hospital of Harbin Medical University, Harbin, 150001 People’s Republic of China; 2 Department of Magnetic Resonance, The First Affiliated Hospital of Harbin Medical University, Harbin, 150001 People’s Republic of China; 3 Department of Pathology, The First Affiliated Hospital of Harbin Medical University, Harbin, 150001 People’s Republic of China

**Keywords:** Nuciferine, Glioblastoma, SOX2-AKT/STAT3-Slug signaling pathway, EMT

## Abstract

**Background:**

Nuciferine (NF), extracted from the leaves of *N. nucifera Gaertn*, has been shown to exhibit anti-tumor and anti-viral pharmacological properties. It can also penetrate the blood brain barrier (BBB). However, the mechanism by which NF inhibits glioblastoma (GBM) progression is not well understood. We aimed to determine the anti-tumor effect of NF on GBM cell lines and clarify the potential molecular mechanism involved.

**Methods:**

U87MG and U251 cell lines were used in vitro to assess the anti-tumor efficacy of NF. Cytotoxicity, viability, and proliferation were evaluated by MTT and colony formation assay. After Annexin V-FITC and PI staining, flow cytometry was performed to evaluate apoptosis and cell cycle changes in NF-treated GBM cells. Wound healing and Transwell assays were used to assess migration and invasion of GBM cells. Western blot analysis, immunofluorescence staining, immunohistochemistry, and bioinformatics were used to gain insights into the molecular mechanisms. Preclinical therapeutic efficacy was mainly estimated by ultrasound and MRI in xenograft nude mouse models.

**Results:**

NF inhibited the proliferation, mobility, stemness, angiogenesis, and epithelial-to-mesenchymal transition (EMT) of GBM cells. Additionally, NF induced apoptosis and G2 cell cycle arrest. Slug expression was also decreased by NF via the AKT and STAT3 signaling pathways. Interestingly, we discovered that NF affected GBM cells partly by targeting SOX2, which may be upstream of the AKT and STAT3 pathways. Finally, NF led to significant tumor control in GBM xenograft models.

**Conclusions:**

NF inhibited the progression of GBM via the SOX2-AKT/STAT3-Slug signaling pathway. SOX2-targeting with NF may offer a novel therapeutic approach for GBM treatment.

**Electronic supplementary material:**

The online version of this article (10.1186/s13046-019-1134-y) contains supplementary material, which is available to authorized users.

## Background

Glioblastoma (GBM) is the most common and aggressive malignant intracranial tumor [1]. Despite multimodal treatment options including surgical resection, chemotherapy, and radiotherapy, the median survival is typically less than 16 months [2, 3]. Recurrence induced by invasive growth and radio−/chemo-resistance has been considered a principal fatal factor that contributes to the poor prognosis. Elucidating the key mechanisms of invasive growth and radio−/chemo-resistance is critical for identifying effective chemotherapeutic drugs in GBM.

Epithelial-to-mesenchymal transition (EMT)—a multistep biological process that converts polarized epithelial cells into mesenchymal cells—is proven to be closely related to tumor migration and invasion. In addition, several studies have demonstrated that EMT is crucial for the proliferation, anti-apoptosis, stemness, and tumor radio−/chemo-sensitivity of cancer cells [4–6]. Among them, stemness of cancer cells has been demonstrated to be responsible for drug resistance. Notably, the EMT process is precisely manipulated by a group of transcriptional factors called EMT regulatory factors, namely, Snail, Slug, Twist, ZEB1, and ZEB2. These master regulators of EMT may also control the aforementioned EMT-related migration, invasion, proliferation, anti-apoptosis, stemness, and tumor radio−/chemo-sensitivity of cancer cells [7–9]. Previous studies showed that EMT regulatory factors modulate these processes by dominating the expression of corresponding markers in cancer cells. Intriguingly, these markers can also regulate the EMT regulatory factors through methods that are dependent or independent on key cell signaling pathways. Ultimately, these factors form highly nodal networks, which make them appealing anti-cancer therapeutic targets.

Sex determining region Y (SRY)-box 2 (*SOX2*) is an intron-less single-exon gene, located on chromosome 3q26.3-q27, and encodes a 317-amino acid protein. As a member of the SOX family of transcription factors, SOX2 regulates multiple stages of mammalian development [10, 11]. In GBM, *SOX2* is a stemness-related gene and has been shown to regulate tumor-initiating and drug-resistant properties in GBM stem cells (GSCs) [12]. GBM cells with elevated expression of *SOX2* show more resistance to temozolomide (TMZ), while its inhibition makes glioma cells more sensitive to this first-line chemotherapy drug [13]. SOX2 has implicitly been demonstrated to regulate EMT in GBM. Taken together, these data suggest that complex regulatory relationships exist between SOX2 and EMT regulatory factors. Therefore, targeting SOX2 activity may provide a novel and attractive approach to treat GBM, particularly with regard to stemness and drug resistance.

Natural metabolites and phytochemicals from plants exhibit low toxicity and therefore receive more attention given their pharmacological effects in the treatment of cancers [14, 15]. Numerous studies have demonstrated that these natural products can inhibit tumorigenesis, proliferation, metastasis, and other hallmark functions of human cancer cells. These natural derivatives have become new treatment strategies for cancers because of their promising chemotherapeutic and chemopreventive properties. Among them, plant alkaloids such as harringtonine, camptothecin, matrine, and vincristine are considered rich sources of anticancer drugs. Nuciferine (NF), an alkaloid extracted from *Nelumbo nucifera Gaertn*, has been proven to have a variety of biological effects including stimulating insulin secretion [16], and reducing atherosclerosis by inhibiting proliferation and migration of vascular smooth muscle cells [17]. In vivo studies have shown that NF exhibits beneficial effects on HIV, melanoma, non-small cell lung cancer, non-alcoholic fatty liver disease, and colorectal cancer [18–22]. Importantly, NF was found to have anti-tumor effects against human neuroblastoma SY5Y cells, and can penetrate the blood-brain barrier (BBB) [22, 23]. This suggests that NF may have therapeutic effects on intracranial tumors such as GBM. Our study aims to evaluate the anti-GBM effects of NF and explore its potential molecular mechanisms of action.

## Materials and methods

### Cells and reagents

The GBM cell lines (U87MG and U251), human umbilical vein endothelial cells (HUVECs), human renal tubular epithelial cells (HK-2), and human normal hepatic cells (LO2) were originally purchased from the American Type Culture Collection (Manassas, VA, USA). Hepatocellular carcinoma cell lines (HepG2, Huh7, and HCCLM3); breast cancer cell lines (MDA-MB-231 and MCF7); and cervical carcinoma cell lines (HeLa) were donated by the Central Laboratory of the First Affiliated Hospital of Harbin Medical University (Harbin, China). HUVECs, LO2 cells, U87MG cells, U251 cells, HepG2 cells, Huh7 cells, and HCCLM3 cells were cultured in Dulbecco’s Modified Eagle’s Medium (DMEM; GE Healthcare, Chicago, IL, USA) supplemented with 10% fetal bovine serum (FBS) at 37 °C in a standard humidified incubator under 5% CO_2_ atmosphere. In addition, HK-2 cells, MDA-MB-231 cells, MCF7 cells, and HeLa cells was cultured in RPMI 1640 medium (GE Healthcare) with 10% FBS. NF (cat. no. N115702) was supplied by Aladdin Industrial Corporation (Shanghai, China). NF was dissolved in methanol as a 56 mmol/L stock solution. Primary antibodies used to detect STAT3, ERK, p-AKT, p-STAT3 and p-ERK were all purchased from Cell Signaling Technology (Danvers, MA, USA). Primary antibodies for detecting E-cadherin, N-cadherin, Vimentin, HIF1A, VEGFA, AKT, CD133, SOX2, CyclinB1, CDC2, Bax, Bcl-2, Snail, Slug, Twist, ZEB1, ZEB2, and β-actin were supplied by Proteintech Group (Wuhan, China). The secondary antibodies were HRP-conjugated AffiniPure goat anti-rabbit IgG and HRP-conjugated AffiniPure Goat anti-mouse IgG (Proteintech Group).

### MTT assay

MTT assay was performed to assess the cytotoxicity of NF. Briefly, 5000 cells/well were cultured in different doses of NF (0–180 μM) for different time periods (0–72 h) in a 96-well plate. After staining with MTT solution (5 mg/mL, 20 μL/well, 4 h) (Sigma-Aldrich, Merck KGaA, Darmstadt, Germany), 150 μl of DMSO was added to each well to solubilize the formazan crystals. Absorbance at 490 nm was then measured by a microplate reader (ELx808, BioTek Instruments, Winooski, VT, USA). The inhibition rate of cellular proliferation was calculated using the equation: inhibition rate (%) = [1-A490 (test)/A490 (blank)] × 100%. The experiments were repeated three times.

### Plate colony-forming assay

Briefly, 1000 GBM cells were seeded in a culture dish measuring 6 cm in diameter for 24 h. Then, different doses of NF (0–90 μM) were used to treat the GBM cells for an additional 3 h, after which the supernatant was replaced by DMEM containing 10% FBS. After culturing for 2 weeks, the cells were fixed with methanol and stained with 0.5% crystal violet. Cell colonies were counted under a light microscope. The experiments were repeated three times.

### Cell cycle assay

After being treated with NF (50 μM) for 48 h, GBM cells were harvested and fixed with 75% ethanol for 12 h. The fixed cells were digested and stained using RNase and propidium iodide, respectively. Cell cycle was accessed with flow cytometry (BD Biosciences, Franklin Lakes, NJ, USA). The experiments were repeated three times.

### Apoptosis assay

GBM cells were plated overnight for adhesion to 6-well plates at a concentration of 2.5 × 10^5^ cells/well. After treating with different doses of NF (0–150 μM) for 24 and 48 h, GBM cells were stained with Annexin V-FITC/PI Apoptosis Detection kit (4A Biotech, Beijing, China). Flow cytometry was used to quantify the apoptotic cells. The experiments were repeated three times.

### Wound-healing assay

The wounds were created by scratching a confluent monolayer of GBM cells with a pipette tip, which were then exposed to different doses of NF (0–30 μM) for 24 h. Images were obtained at 0 h, 24 h, and 48 h with a microscope to analyze movement of the cells to close the wound. ImageJ software (National Institutes of Health, Bethesda, MD, USA) was used to analyze the migration distance. The experiments were repeated three times.

### Transwell assay

The migration and invasion of GBM cells were assessed by transwell chambers (8-μm pore size, Corning, Tewksbury, USA). GBM cells seeded in 6-well plates were cultivated with different doses of NF (0–30 μM) for 24 h. For transwell assay, the lower compartment of the chamber was filled with medium containing 10% FBS, while the corresponding upper chamber was seeded with pre-treated GBM cells (5 × 10^4^ cells per well) suspended in serum-free medium (200 μl). For the invasion assay, the upper transwell chambers were covered with 50 μl of Matrigel (BD Biosciences, Franklin Lakes, NJ, USA) to form a continuous membrane. After incubation for 24–48 h, migratory or invasive cells were stained with 0.5% crystal violet and analyzed under a light microscope. The experiments were repeated three times.

### Western blot analysis

GBM cells were treated with different doses of NF (0–150 μM) for 48 h, and then lysed using RIPA buffer (Beyotime, Shanghai, China). After centrifugation at 12,000 rpm for 10 min, the supernatants were transferred to a new tube. The protein concentration was measured using bicinchoninic acid (BCA) method. The proteins were separated by SDS-PAGE and then transferred onto PVDF membranes (Millipore, Bedford, MA). After being blocked with 5% non-fat milk/TBST, the membrane was incubated with the corresponding primary antibody and HRP-conjugated secondary antibody. Protein signals were assessed using enhanced chemiluminescence (Thermo Fisher Scientific, Waltham, MA, USA). The experiments were repeated three times.

### Immunofluorescence

GBM cells in a 24-well plate were exposed to NF (30 μM) for 48 h and fixed with 4% paraformaldehyde. After being incubated with blocking solution (0.1% Triton-100 in normal goat serum), GBM cells were then incubated with a primary antibody and then a fluorescein (FITC)-conjugated secondary antibody for each protein of interest. Nuclei of GBM cells were stained with DAPI before images were acquired using a fluorescence microscope. The experiments were repeated three times.

### Bioinformatics analysis

GEPIA (http://gepia.cancer-pku.cn/index.html) was employed for conducting tumor/normal differential expression analysis, patient survival analysis, and multiple gene comparison analysis. The Human Protein Atlas (http://www.proteinatlas.org) was used to determine the distribution of SOX2, CD44, and Nestin proteins in the cancer cells and to compare the SOX2 protein level in normal brain and GBM tissues, as detected by a SOX2 antibody (CAB010648).

### Transient transfection of siRNAs

*SOX2* silencing was achieved via transfection of specific siRNAs (Genepharma, Shanghai, China), with the help of Lipofectamine 2000 (Invitrogen, Carlsbad, California, USA). The sequences of the siRNAs are shown in Additional file 1: Table S1.

### Animal tumor model and treatments

BALB/c nude mice (4–5 weeks old) were obtained from Charles River Japan (Beijing, China) and maintained in a pathogen-free environment. The design of the animal experiment was reviewed and approved by the Committee on the Use of Live Animals in Teaching and Research of the Harbin Medical University (Harbin, China). After anesthetizing with an intraperitoneal injection of pentobarbital sodium (1%; 5 mL/kg), BALB/c nude mice were subcutaneously inoculated with U251 cells in the left flank. After 2 weeks, U251 tumor-bearing nude mice with tumor sizes of approximately 200 mm^3^ were randomly assigned to two groups (*n* = 5, each group): control and NF treatment. Mice in the NF treatment group were intraperitoneally injected with NF at a dose of 15 mg/kg, once a day for a total of 2 weeks. Mice in the control group were intraperitoneally injected with isometric PBS. The tumor changes were monitored by ultrasonic imaging (USI), magnetic resonance imaging (MRI), and pathology. The tumor volume was calculated using the formula, V = length × width^2^/2.

### Ultrasonic imaging

B-mode ultrasonography, color Doppler flow imaging (CDFI), color power angiography (CPA), and ultrasonic elastosonography (USE) of Philips iU Elite Ultrasound System (Philips Healthcare, Amsterdam, The Netherlands) were used to estimate tumor growth, angiogenesis, micro-angiogenesis, and degree of hardness, respectively.

### Magnetic resonance imaging

MRI was performed on a Philips Achieva 3.0 T TX MRI System to evaluate changes in tumor growth and signal intensity. The specific imaging sequences were T1WI, T2WI, T2-FLAIR, and T2-SPIR, which are widely used in clinical craniocerebral imaging.

### Immunohistochemistry (IHC)

Tumors from U251 tumor-bearing nude mice were fixed with formaldehyde and embedded in paraffin. Subsequently, the tissue samples were sectioned for immunostaining with antibodies against target proteins. Immunohistochemical staining was conducted by employing the streptavidin-peroxidase complex. Images were then captured using a light microscope.

### Statistical analysis

IBM SPSS 22.0 software (Armonk, NY, USA) was used to perform statistical analysis. Data are shown as mean ± standard deviation (SD). Difference between the groups was analyzed either by Student’s *t*-test or ANOVA. *P* < 0.05 was considered statistically significant.

## Results

### Cytotoxicity of NF in GBM cells and non-cancer cells

MTT assays were performed to determine the cytotoxicity of NF (100 μM, 48 h) in four types of cancers with high mortality or morbidity, including breast cancer (MDA-MB-231 and MCF7); hepatocellular carcinoma (HepG2, Huh7, and HCCLM3); cervical carcinoma (HeLa); and GBM (U87MG and U251). NF showed obvious growth inhibitory effects in HCCLM3, U87MG, and U251 cells (Fig. 1a). Due to the significant decrease in GBM cell viability induced by NF, further dose-dependent viability studies were performed using a wide range of NF concentrations (0–180 μM) over the course of 24, 48, and 72 h. The results showed that NF could effectively inhibit the growth of GBM cells in a dose- and time-dependent manner (Fig. 1b and c, Additional file 2: Figure S1). Using Probit regression analysis, we observed 50% inhibitory concentration values (IC50) of NF in U87MG and U251 cells of approximately 72.3 μM and 59.9 μM at 48 h, respectively. Notably, NF exhibited minimal cytotoxicity on normal human cells (HUVECs, LO2, and HK2) (Additional file 2: Figure S2). Colony formation is a process by which a single cell proliferates into a cell cluster. Thus, colony formation rate, to some extent, may reflect stemness, where a single tumor cell can repopulate a bulk tumor. Treatment with NF reduced the ability of GBM cells to form colonies (Fig. 1d), suggested a deficiency in stemness. This observation was further supported by an NF-induced decrease in the stemness marker CD133 (Fig. 1e). Deregulation of the cell cycle is a fundamental mechanism of infinite and rapid proliferation of cancer cells. In this study, cell cycle analysis by flow cytometry demonstrated that NF treatment resulted in G2 phase cell cycle arrest in GBM cells (Fig. 1f, g and h). To elucidate the underlying mechanism of G2 phase arrest induced by NF, we analyzed cell cycle regulatory proteins by western blot. As shown in Fig. 1e, the expression level of CDC2 was decreased following NF treatment in a dose- dependent manner, while an increased expression of CyclinB1 was also observed.

**Fig. 1:** Effect of NF on the proliferation of GBM cells. **a** Different cancer cell lines were treated with NF (100 μM, 48 h), and then the percentages of viable cells were determined using MTT assay. *P < 0.05, **P < 0.01 vs. control group. **b** and **c** U87MG and U251 cells were treated with NF (0–180 μM, 0–72 h) and the inhibition rates were determined using MTT assay. **d** Colony formation assay was used to confirm the growth inhibitory effect of NF (0–90 μM, 3 h). **e** CDC2 and CD133 were decreased, and CyclinB1 was increased in GBM cells treated with NF (0–150 μM, 48 h), the expression of the indicated factors was examined by western blot. β-actin was used as the loading control. **f**, **g** and **h** Cell cycle assay of U87MG and U251 cells after treatment with NF (50 μM, 48 h). Data are represented as mean ± SD (*n* = 3), **P < 0.01

Cell cycle is a complex process, which is precisely orchestrated by the temporal expression of CDK/cyclin family members [24]. Generally, the expression of CDC2 is increased in G2 phase, and then CDC2 combines CyclinB1 to form the CDC2-CyclinB1 complex, called the maturation promoting factor (MPF) [25]. Activation of the MPF is required for the transition from G2 phase into M phase. The catalytic subunit CDC2 can regulate the activity of MPF through its own phosphorylation and dephosphorylation. After CDC2 binding to CyclinB1, phosphorylation of CDC2 (Thr14, Tyr15, and Thr161) mediated by upstream kinases, including Myt1, WEE1 and CDK7, can repress the activity of MPF. In the late G2 phase, CDC25C phosphatase, a division protein of cell cycle, can dephosphorylate both phospho-Thr14 and phospho-Tyr15 of CDC2, thereby enabling MPF to acquire biological activity and induce mitosis [24, 26]. On the contrary, inactivation of CDC2 can arrest the cell cycle in G2 phase [27]. In addition, Piao et al. also reported that G2 phase arrest was correlated with the downregulation of CDC2 in a study of DYC-279 in the treatment of hepatocellular carcinoma [28]. In conclusion, CDC2 is the critical regulatory factor for the activation of MPF, and its inactivation or reduction can arrest the cell cycle in G2 phase. Therefore, the NF-induced G2 phase arrest observed in this study may be at least partially ascribed to the decreased expression of CDC2 protein, which may reduce the production and activation of MPF.

In addition to CDC2, CyclinB1, as a regulatory subunit of MPF, can regulate the activity of MPF through its own synthesis and degradation. This process may be illustrated as follows: first, CyclinB1 is synthesized during the late S through G2 phases, then it forms MPF with CDC2 to promote the transition from G2 phase into M phase [29]; second, at the end of the G2/M transition, CyclinB1 is quickly ubiquitinated and degraded by the proteasome complex, resulting in a decrease in the content and activity of MPF [30, 31], which is required for cytokinesis and univalent chromosome movement to exit from mitosis [32–34]. In this scenario, regardless of the decrease in initial CyclinB1 synthesis, or the later reduction in CyclinB1 degradation, they all have the potential to induce G2 cell cycle arrest. Based on this, the unconventional increase in CyclinB1 in G2 arrested cells that has been reported by several studies, may be partially explained by the reduction in CyclinB1 degradation [28, 35, 36]. Therefore, in our study, it is probably that the incremental expression of CyclinB1 is also associated with the reduction of its degradation, which keeps GBM cells from exiting mitosis, hence contributing to NF-induced G2 arrest.

In summary, we can conclude that NF may restrain the initial synthesis of CDC2, but not CyclinB1, which then reduce the content and activity of MPF, and subsequently in G2 cell cycle arrest. Additionally, the reduction in CyclinB1 degradation at the later stage, may impede the termination of mitosis, and further aggravate G2 cell cycle arrest.

### NF induced apoptosis in GBM cells

Exposure to NF resulted in distinct morphological changes in GBM cells, which became rounder and smaller in comparison to controls. NF-treated GBM cells also separated from the bottom of the culture plate. These morphological changes in GBM cells indicated that NF-induced growth inhibition could also be attributed to apoptosis in addition to the anti-proliferative effect. As expected, NF (48 h) induced overt dose-dependent apoptosis in U87MG and U251 cells (Fig. 2a and b). Additionally, statistical analysis indicated that the proportion of apoptotic cells after the 150-μM NF treatment was 10.28- and 11.53-fold higher in comparison to the control group in U87MG and U251 cells, respectively. Since apoptosis is a biological process with distinct early and late stages, U87MG and U251 cells were then treated with NF for 24 h (shorter treatment). The result showed that NF (24 h) also induced significant dose-dependent apoptosis, and the proportion of early apoptotic cells was increased in comparison to the proportion at 48 h (Additional file 2: Figure S3). Western blot analysis also showed increased Bax expression (pro-apoptosis marker) and decreased Bcl-2 expression (anti-apoptosis marker) in NF-treated GBM cells, suggesting that NF-induced apoptosis is being driven by the intrinsic apoptosis pathway (Fig. 2c).

**Fig. 2:** Apoptosis of GBM cells after treatment with NF (0–150 μM, 48 h). **a**, **b** Cell apoptosis assay of GBM cells after treatment with NF at different concentrations (0–150 μM, 48 h). **P < 0.01. **c** NF (0–150 μM, 48 h) suppressed Bcl-2 and Bax in GBM cells and the expression of the indicated factors was examined by western blot. β-actin was used as the loading control

### NF inhibited motility of GBM cells

In addition to inducing apoptosis in cancer cells, many chemotherapies also have the ability to impede tumor cell motility. Therefore, we used wound-healing assays to assess the inhibitory effect of NF on the motility of GBM cells. We used lower NF concentrations (0–30 μM) in order to delineate the effect of motility without impairing viability. NF impeded the motility of GBM cells in a dose-dependent manner in comparison to control NF-free cells, which were able to move and repair the scratch (Fig. 3a and b). Similarly, transwell assays also showed dose-dependent decreases in migration and invasion of NF-treated GBM cells (Fig. 3c and d).

**Fig. 3:** Mobility of GBM cells after NF treatment. **a**, **b** Wound-healing assay of GBM cells after treatment with NF (0–30 μM, 24 h) at non-lethal concentrations. **c**, **d** Migration and invasion assay of GBM cells after treatment with NF (0–30 μM, 24 h) at non-lethal concentrations. Compared with the control group (0 μM NF), **P < 0.01

Another key hallmark of cancer cells is their ability to grow new vasculature to increase blood supply and to help facilitate metastatic spread. Therefore, we investigated the effect of NF on angiogenesis in GBM cells. Western blot analysis of key angiogenic factors HIF1A and VEGFA revealed that NF treatment resulted in decreased HIF1A and VEGFA levels in GBM cells (Additional file 2: Figure S4).

### NF inhibited EMT in GBM cells

In addition to being important for migration and invasion, EMT has also been shown to be a pivotal mechanism in cancer cells for enhanced proliferation, stemness, angiogenesis, and anti-apoptotic properties [4, 5]. Therefore, we determined the effect of NF on EMT in GBM cells, by evaluating the expression of key EMT biomarkers, such as E-cadherin, N-cadherin, and Vimentin. Western blot assays showed that the expression of mesenchymal markers, N-cadherin and Vimentin, was decreased with increasing doses of NF, whereas the expression of the epithelial marker E-cadherin was increased (Fig. 4a and b). Immunofluorescence assays confirmed increased E-cadherin and decreased Vimentin expression in U87MG and U251 cells after NF treatment (Fig. 4c). These changes in N-cadherin, Vimentin, and E-cadherin indicated that a mesenchymal-to-epithelial transition (MET) occurred after NF treatment, which is the reverse process of EMT.

**Fig. 4:** NF repressed EMT in U87MG and U251 cells. **a**, **b** The expression of E-cadherin, N-cadherin, and Vimentin after NF treatment (0–150 μM, 48 h). *P < 0.05, **P < 0.01 vs. control group. **c** Immunofluorescence assay (scale bar: 200 μm) of E-cadherin and Vimentin after NF treatment (30 μM, 48 h)

### Slug expression was inhibited by NF in GBM cells

The expression levels of EMT regulatory factors in GBM, such as Snail, Slug, Twist, ZEB1, and ZEB2, were estimated by western blot assays. The results showed that the expression of Slug was significantly decreased by NF in U87MG and U251 cells in a dose-dependent manner (Fig. 5a). However, the expression of Snail, Twist, ZEB1, and ZEB2 were only moderately changed. Immunofluorescence assay confirmed the decrease in Slug in NF-treated U87MG and U251 cells (Fig. 5b). Slug has been shown to be involved in several tumorigenic processes in cancers such as breast, prostate, pancreas, and GBM [37, 38]. This includes EMT, proliferation, cell cycle, stemness, angiogenesis, and anti-apoptosis [39]. These results suggest that NF may exert the aforementioned functions by suppressing Slug.

**Fig. 5:** Expression of EMT regulatory factors and signaling pathway after NF treatment in GBM cells. **a** After NF treatment (0–150 μM, 48 h), Slug was decreased in a dose-dependent manner. *P < 0.05, **P < 0.01 vs. control group (0 μM NF). **b** Immunofluorescence assay (scale bar: 200 μm) of Slug after NF treatment (30 μM, 48 h) in U87MG and U251 cells. **c** Western blot assay of main protein expression of signaling pathways after NF treatment (0–150 μM, 48 h). **P < 0.01 vs. control group (0 μM NF)

### NF inhibited two vital signaling pathways of GBM cells

The pivotal factors of three vital cell signaling pathways in GBM cells were detected by western blot assays, including AKT, ERK1/2, STAT3 and their corresponding phosphorylated forms (p-AKT, p-ERK1/2, p-STAT3). The results revealed that p-AKT and p-STAT3 expression were notably reduced by NF in a dose-dependent manner (Fig. 5c). Nevertheless, total AKT and STAT3 expression showed no statistical difference. Moreover, no significant changes were found in ERK1/2 and p-ERK1/2.

### SOX2 is a therapeutic target of GBM cells

By querying online bioinformatic databases, we identified that the mRNA expression levels of *SOX2, CD44*, and *Nestin* were the most significantly altered stemness makers in GBM tissues (Additional file 2: Figure S5). By using the Human Protein Atlas (HPA), we found that SOX2 protein was principally distributed in the nuclei, CD44 was limited to the plasma membrane and Golgi apparatus, and Nestin to the intermediate filaments (Fig. 6a, Additional file 2: Figures S6 and S7). The median expression of *SOX2* was higher in the brain tissue than in other organs (Fig. 6d). Moreover, GBM/normal differential expression analysis revealed that the expression of *SOX2* in GBM tissues was higher than that in normal brain tissues, regardless of the protein level or mRNA level (Fig. 6b and c). The mRNA expression of *SOX2* in GBM was the second highest among 31 types of tumors (Fig. 6e, Additional file 1: Table S2), while LGG (lower grade gliomas) ranked first. However, there was no significant association between high expression of *SOX2* and overall survival (OS) or disease-free survival (DFS) in GBM patients (Additional file 2: Figure S8).

**Fig. 6:** SOX2 as a therapeutic target of GBM. **a** Subcellular localization of SOX2 (The Human Protein Atlas). **b** Protein level of SOX2 in normal tissue and GBM (The Human Protein Atlas). **c** mRNA level of *SOX2* in normal tissue and GBM (GEPIA). **d** Median expression in tumor (red) and normal (green) samples in the body map (GEPIA). **e** mRNA level of *SOX2* in 31 different kinds of tumors (GEPIA). **f** Western blot assay of SOX2 after siRNA transfection using control siRNA RNAi-NC, or *SOX2-*targeting siRNAs RNAi1, RNAi2, and RNAi3 in U87MG and U251 cells. **g** Western blot assay of SOX2 after treatment with different concentrations of NF (0–150 μM, 48 h) in GBM cells. **h** siRNA-mediated knockdown of *SOX2* in GBM cells led to significant inhibition of p-AKT, p-STAT3, and Slug. **i** Immunofluorescence assay (scale bar: 200 μm) of SOX2 after treatment with NF (30 μM, 48 h) in U87MG cells . **j** Immunohistochemical analysis of SOX2 expression after treatment with NF (15 mg/kg, once a day for a total of 2 weeks) in the U251 xenograft tumors (original magnification: × 400, scale bar: 100 μm). **k** Insight into a SOX2-dependent mechanism of NF-induced (100 μM, 48 h) inhibition of cell proliferation in U251 cells by MTT assay. *P < 0.05, **P < 0.01 vs. control group

In this study, we found RNAi1 and RNAi2 could effectively downregulate the expression of *SOX2* (Fig. 6f). In addition, western blot assays showed that decreased levels of p-AKT, p-STAT3, and Slug after siRNA-mediated knockdown of *SOX2* (Fig. 6h). Additionally, no significant changes were observed in the expression of total AKT, STAT3, ERK1/2, and p-ERK1/2. These results indicated that SOX2 may be upstream of p-AKT, p-STAT3, and Slug.

SOX2 expression was decreased after treatment with different NF concentrations (Fig. 6g, Additional file 2: Figure S9). Immunofluorescence assays confirmed decreased SOX2 in NF-treated U87MG and U251 cells (Fig. 6i, Additional file 2: Figure S10). The results of IHC showed that SOX2 expression was decreased in tumor tissues in the NF treatment group (Fig. 6j).

Lastly, to ascertain whether SOX2 mediated the therapeutic functions of NF, rescue experiments were performed. These revealed that NF had a greater therapeutic effect than *SOX2-*knockdown alone. Additionally, siRNA-mediated suppression of *SOX2* in GBM cells resulted in a partial reversal of NF-induced growth inhibition (Fig. 6k, Additional file 2: Figure S11). These results suggest that NF-induced cell growth of GBM cells may be mediated by a SOX2-dependent mechanism.

### NF inhibited the growth of GBM xenograft tumors in nude mice

Using BALB/c nude mice, we established a U251 xenograft tumor model to evaluate the anti-tumor activity of NF in GBM in vivo. NF significantly suppressed tumor growth, as tumor weights and sizes in the NF treatment group were obviously smaller than those of the control group on day 14 (Fig. 7a–d). We then further demonstrated that tumor growth was suppressed by NF in a dose-dependent manner (Additional file 2: Figure S12). Western blot results also revealed that AKT, p-AKT, STAT3, p-STAT3, SOX2, Slug, N-cadherin, Vimentin, CD133, Bcl-2, CDC2, HIF1A, and VEGFA protein expression in excised xenograft tumors were notably decreased in a dose-dependent manner, while E-cadherin was increased (Additional file 2: Figure S13). IHC was employed to evaluate the protein expression of representative tumor progression markers in the xenograft tumors harvested from the two groups. The results showed that Ki67, CDC2, Bcl-2, HIF1A, and N-cadherin were decreased in the NF-treated group in comparison to controls (Fig. 7e). Noninvasive imaging can provide abundant information about tumor progression and allow for the assessment of multiple parameters that are inaccessible by the naked eye. Furthermore, the change in total gene expression may be reflected by noninvasive imaging [40, 41]. We employed USI (B-mode, CDFI, CPA, and USE) and MRI (T1WI, T2WI, T2-FLAIR, and T2-SPIR) to monitor the internal changes in the tumors. In comparison to the control group, tumor size, angiogenesis, and hardness index were all decreased in the NF treatment group (Fig. 7f). MRI images showed similar results as B-mode ultrasound with respect to tumor growth (Fig. 7g). H&E staining confirmed decreased angiogenesis in the NF treatment group (Additional file 2: Figure S14). To determine if NF caused any adverse effects in internal organs, we harvested the heart, liver, spleen, lung, and kidney of the mice in the two groups. H&E staining showed that NF treatment did not induce obvious necrosis in comparison to the controls (Additional file 2: Figure S15).

**Fig. 7:** NF inhibited the growth of U251 xenograft tumors in nude mice. **a-d** U251 cells were subcutaneously injected into the mouse left flank to establish xenograft models. After NF treatments (15 mg/kg, once a day for a total of 2 weeks), all mice were observed, and the tumor weight and volume were measured and compared. **P < 0.01 vs. control group. **e** Expression of Ki67, CDC2, Bcl-2, HIF1A, and N-cadherin in xenograft tumors were analyzed by immunohistochemistry (original magnification: × 400, scale bar: 100 μm). **f** Ultrasonography evaluation included B-mode, CDFI, CPA, and USE. **g** T1WI, T2WI, T2-FLAIR, and T2-SPIR imaging of tumors by MRI

## Discussion

GBM is the most common and malignant brain neoplasm. Current standard treatments of maximal resection followed by adjuvant chemotherapy and radiotherapy, are powerless to ameliorate the clinical outcome of GBM patients [2, 3]. Recurrence induced by EMT-related invasive growth and radio−/chemo-resistance is a principal fatal factor that contributes to the poor prognosis.

The tremendous medicinal potential of lotus plants has been documented by Ayurveda and traditional Chinese medicine. In several pre-clinical studies, lotus extracts have displayed remarkable anticancer effects. As an aporphine alkaloid extracted from the lotus leaf, NF has shown potent suppressive effects in neuroblastoma, melanoma, non-small cell lung cancer (NSCLC), and colorectal cancer [19, 20, 22]. Nevertheless, the anti-GBM activity of NF is unknown. For the first time, our study showed that NF can inhibit proliferation, invasion, EMT, stemness, and angiogenesis, and can induce apoptosis in GBM.

Comparing and analyzing differences in molecular characteristics between cancer cells with high sensitivity and low sensitivity to a specific chemotherapeutic drug has been recognized as a classical method for identifying drug therapeutic targets. Accordingly, we detected the cytotoxicity of NF in several representative cancer cell lines with high mortality or morbidity, and the results showed that NF displayed prominent therapeutic effects on cancer cells with strong mesenchymal properties, specifically HCCLM3, U87MG, and U251 cells. The potency of the anti-tumor effect of NF in GBM cell lines (U87MG and U251) was intriguing to us and has since been the focus of our research. GBM is a malignancy with high mesenchymal levels, which may allow for the clinical application of NF in this disease indication. Based on this hypothesis, our study discovered that the expression of mesenchymal markers N-cadherin and Vimentin was remarkably decreased, while the expression of the epithelial marker E-cadherin was increased after NF treatment. These results suggest that NF can promote MET to reduce the mesenchymal phenotype of GBM cells. An enhanced mesenchymal phenotype is often accompanied by stronger metastatic, proliferative, stemness, anti-apoptotic, and angiogenetic abilities, which are co-regulated by EMT regulatory factors [4]. Therefore, the stemness marker (CD133), G2 phase marker (CDC2), anti-apoptosis marker (Bcl-2), and angiogenesis markers (HIF1A and VEGFA) were also detected and shown to be reduced with a decrease in the mesenchymal phenotype of GBM cells after NF treatment. These results indicated that NF can inhibit the proliferation, stemness, angiogenesis, and anti-apoptotic effects at the molecular level.

Inferring from the results above, we then evaluated the expression of upstream regulators of the aforementioned markers, namely the five representative EMT regulatory factors: Slug, Snail, Twist, ZEB1, and ZEB2. Slug emerged as the best candidate because it was unanimously and remarkably suppressed by NF in GBM cells. In addition, Yang et al. demonstrated that Slug can accelerate proliferation, migration, invasion, and angiogenesis in GBM [42]. These studies have summarily indicated that NF may exert anti-GBM effects by regulating Slug expression. Subsequently, the AKT and STAT3 signaling pathways that are the upstream signaling pathways of Slug [43–45] were shown to be suppressed by NF. Notably, the AKT signaling pathway has been identified as one of the three central cell signaling pathways of GBM by The Cancer Genome Atlas (TCGA), based on a thorough and comprehensive genomic characterization of 206 human GBM samples [46]. Specifically, the suppression of the AKT signaling pathway is fatal for GBM cells. This may be one pivotal reason why NF exhibits impressive anti-GBM functions.

The AKT and STAT3 signaling pathways can manipulate EMT regulatory factors to activate the genes related to GBM stemness directly or indirectly, such as *CD133, CD44, Oct4, SOX2, Nanog, ALDH1A1, Olig2,* and *Nestin* [47]. As a result, GBM cells with persistent stemness can acquire detrimental chemo- and radio-resistance. Among these stemness markers, *SOX2, CD44,* and *Nestin* were highly expressed in GBM tissues (Additional file 2: Figure S5). Recent studies investigating the subcellular localization of stemness markers demonstrated that the reprogramming activity of these markers was limited to the cell nucleus rather than the cytoplasm [48]. Using the HPA, we identified that SOX2 protein was primarily distributed in the cell nucleus, CD44 was limited to the plasma membrane and Golgi apparatus, and Nestin to the intermediate filaments. In 2006, Yamanaka and Takahashi published a seminal study, which demonstrated that differentiated somatic cells can be induced to become pluripotent embryonic stem cells. They also discovered that the transcription factors SOX2, OCT4, KLF4, and c-MYC were adequate for induction of pluripotency in differentiated cells, leading to the generation of induced pluripotent stem cells [49]. This research highlighted the momentous status of SOX2 in maintaining the stemness of stem cells and driving differentiated cells to morph into stem cells. SOX2 is overexpressed in several malignant neoplasms, and the highest expression was found in gliomas (GBM and LGG) (Fig. 6e). The association of SOX2 overexpression and low OS and DFS has also been demonstrated using independent cohorts of GBM patients [13]. AKT and STAT3 signaling pathways and Slug have been shown to regulate SOX2 in previous studies. In our study, we observed that *SOX2* knockdown downregulated the expression of p-AKT, p-STAT3, and Slug. Thus, positive feedback relationships were established between SOX2, AKT, STAT3 and Slug. Simultaneously, these results implied that SOX2 was involved in more than boosting or maintaining the activity of stem cells. In that, it may also contribute to the functional roles of the AKT and STAT3 signaling pathways and Slug through dominating the SOX2-AKT/STAT3-Slug signaling pathway. The SOX2-AKT/STAT3-Slug signaling pathway may exert crucial effects in many biological functions of GBM cells (stem and non-stem cells), suggesting that this may be a crucial node for therapeutic targeting. On account of the inhibitory effect of NF on multiple components of the SOX2-AKT/STAT3-Slug signaling pathway, we then revealed that NF could inhibit the protein expression of SOX2 using western blot and immunofluorescence assays in GBM cells. These results demonstrated that NF could eliminate GBM by suppressing the SOX2-AKT/STAT3-Slug signaling pathway and may prevent the occurrence of chemo- and radio-resistance mediated by stemness (Fig. 8).

**Fig. 8:** NF chemical structure and the inhibitory mechanism of action in GBM. **a** Chemical and 3D structure of NF. **b** Schematic presentation of the mechanism underlying NF-induced inhibition of GBM and relevant molecular mechanism referring to the SOX2-AKT/STAT3-Slug signaling pathway

To further corroborate that the SOX2-AKT/STAT3-Slug signaling pathway mediates the anti-tumor effect of NF on GBM cells, we conducted rescue experiments, in which we observed that the therapeutic effect of NF was better than knockdown of *SOX2* alone. Additionally, adding NF into GBM cells pretreated with si-SOX2 caused no further inhibition (Fig. 6k, Additional file 2: Figure S11). These phenomena illustrate three problems: first, the SOX2-AKT/STAT3-Slug signaling pathway could mediate the therapeutic effect of NF in GBM; second, the SOX2-AKT/STAT3-Slug signaling pathway was the dominant target of NF; and third, NF also had other targets independent of the SOX2-AKT/STAT3-Slug signaling pathway. In previous studies, by employing a traditional Chinese medicine network pharmacology method, Qi et al. confirmed that NF was effective against human neuroblastoma and mouse colorectal cancer by inhibiting PI3K-AKT signaling pathways and reducing IL-1 levels [22]. Moreover, Liu et al. revealed that NF could inhibit the Wnt/β-catenin signaling pathway in non-small cell lung cancer [20]. These data strongly suggest that NF is a multi-target drug. Drugs with multi-targets possess inherent advantages in comparison to single-target inhibitors such as cetuximab, panitumumab, nimotuzumab, and necitumumab. The therapeutic effects of single-target inhibitors are frequently offset by dynamic decoupling, rewiring, or establishment of compensatory signaling pathways in cancer cells [50]. Otherwise, combination strategy of diverse single-target inhibitors usually brings about a host of side effects. Thus, seeking out monotherapy strategies with multiple targets is imperative, and NF is one such potential therapeutic agent.

The capability to penetrate the BBB bestows NF great advantages in GBM therapy. Nevertheless, several studies have indicated that some drugs with the capacity to cross the BBB in pre-clinical studies could not consistently achieve sufficient intratumoral levels to eradicate GBM cells, due in part to poor brain-plasma ratios. For the predicament of drug enrichment, neoteric multifunctional nanoparticles provide a feasible solution for efficient drug delivery [51]. Additionally, the enhanced permeability and retention effect (EPR) of nanoparticles may further augment drug accumulation in tumors through continuous collection of nanoparticles from the circulatory system.

## Conclusions

This study demonstrated that SOX2 has complex mutual regulatory relationships with the AKT and STAT3 signaling pathways, and the EMT regulatory factor Slug. These factors together establish a SOX2-AKT/STAT3-Slug signaling network, which can influence multiple biological functions of GBM cells. Remarkably, NF, as a novel alkaloid chemotherapeutic drug, could inhibit proliferation, migration and invasion (EMT), stemness, and angiogenesis, while possibly promote apoptosis in GBM cells. We further demonstrated that NF exerted these effects primarily via impeding multiple components of the SOX2-AKT/STAT3-Slug signaling pathway. In addition, the minimally cytotoxic effect of NF in normal human cells, prominent BBB permeability, as well as a great potential to be carried by nanomaterials suggest that NF has strong potential for drug development as a therapeutic agent for patients with GBM.

## Additional files

Additional file 1: **Table S1.** The sequences of a control non-targeting siRNA and 3 *SOX2*-targeting siRNAs. **Table S2.** Full names and corresponding abbreviations of 31 different types of tumors. (DOCX 16 kb)

Additional file 2: **Figure S1.** Effect of NF on the viability of U87MG and U251 cells. **Fig S2**. Cell viability of normal human cells after treatment with different concentrations of NF (0–180 μM, 48 h). **Fig S3**. Apoptosis of GBM cells after treatment with NF (0–150 μM, 24 h). **Fig S4**. NF suppressed HIF1A and VEGFA in GBM cells. **Fig S5**. Multiple gene comparisons in GBM: *CD133*, *CD44*, *Oct4*, *SOX2*, *Nanog*, *ALDH1A1*, *Olig2*, and *Nestin* (GEPIA). **Fig S6**. Subcellular localization of SOX2. **Fig S7**. Subcellular localization of Nestin and CD44 (HPA, human protein atlas). **Fig S8**. OS and DFS of GBM patients based on SOX2 expression. **Fig S9**. The expression of SOX2 in GBM cells treated with NF. **Fig S10**. Immunofluorescence assay (Scale bar: 200 μm) of SOX2 after treatment with NF (30 μM, 48 h) in U251 cells. **Fig S11**. Rescue-dependent manner. **Fig S13**. The prot experiment of SOX2 in U87MG cells. **Fig S12**. NF (0, 10, and 15 mg/kg, once a day for a total of 2 weeks) inhibited the growth of U251 xenograft tumors in a dose ein expression in excised xenograft tumors was notably reduced by NF (0, 10, and 15 mg/kg, once a day for a total of 2 weeks) in a dose-dependent manner. **Fig S14**. Pathology changes of angiogenesis. **Fig S15**. No obvious necrosis was found in xenograft mice internal organs. (DOCX 5899 kb)

## Abbreviations

BBB: Blood brain barrier
CDFI: Color Doppler flow imaging
CPA: Color power angiography
DMEM: Dulbecco’s Modified Eagle’s medium
EMT: Epithelial-to-mesenchymal transition
GBM: Glioblastoma
HPA: Human protein atlas
MRI: Magnetic resonance imaging
NF: Nuciferine
USE: Ultrasonic elastosonography
USI: Ultrasonic imaging
